# Application of Watson Visual Perception Model in Nanchang VI Visual Image Recognition Design

**DOI:** 10.1155/2022/3070084

**Published:** 2022-05-24

**Authors:** Jianfeng Huang

**Affiliations:** School of Humanities, Huzhou College, Huzhou 313000, China

## Abstract

To shape a complete city image, it is necessary to find the first characteristic of the city so as to further improve the easy identification of the city image, create a good city image, and make the city more competitive. This paper combines the Watson visual perception model to carry out the visual image recognition design of Nanchang VI to improve the communication effect of the urban VI visual image. Moreover, this paper proposes a video watermarking algorithm based on MPEG-4 encoding using the open-source Xvid codec. In addition, this paper proves that the proposed algorithm has good application value in imperceptibility and robustness through a large number of experiments and data analysis. Finally, this paper verifies the reliability of the method proposed in this paper through the study of multiple sets of data.

## 1. Introduction

In modern society, the improvement of the city image recognition system has become an indispensable and important part in the city image construction. It is widely recognized that the theoretical value and importance of the visual recognition system in the performance of the city's core competitiveness, which penetrates into all fields of politics, economy, culture, and life, also require the cooperation of many interdisciplinary subjects. The introduction of the corporate image recognition system (CIS) theory, for the city image design, is to extract and summarize the creative part of the city image construction with brand effect, so that the many and complex design limitations in various areas of the city can be eliminated. Use the core content of this principle to analyze the specific design problems of urban image identification, break the stereotyped characteristics of traditional urban image design, and reintroduce new life and elements into the design so that people can reunderstand the core elements and elements of urban image design and personality traits. It can also quickly and accurately grasp the specific design direction and method of the visual recognition system, know the principle and operation method of the visual recognition system of the city, accurately grasp the characteristics of the city's personality according to the theoretical guidance of the corporate image recognition system, and formulate accurate complete design action.

For a city with many resources, a city's natural resources, capital resources, human resources, and so on largely determine the speed of urban development, and it is undoubtedly a good development platform for the city [1]. Therefore, the city identification system is a method to help cities better display and express their own development prospects and their own characteristic resources. Moreover, more and better display of these resources urgently requires that the city image design can fully express the comprehensive image display of the city to attract more external attention and recognition, which of course brings more business opportunities [2]. The construction of the city visual identification system can help the city gradually establish a good image system, and a good city image system is an effective external manifestation of the city's competitiveness. Therefore, the establishment of a city image visual identification system with clear personality, strong visual impact, and high recognizability will inevitably become an important asset for the sustainable development of the city. In addition, a relatively complete visual identification system of city image, which is easier to identify and has a brand effect according to the city's own characteristics, is the focus of this study. With the improvement of this system, the city can formulate a more perfect environment, optimize the interaction between various land resource elements, and play a vital role in cultivating the overall sustainable economic environment of the city [3].

This paper combines the Watson visual perception model to carry out the Nanchang VI visual image recognition design, improve the communication effect of the urban VI visual image, and provide a theoretical reference for urban publicity and development.

## 2. Related Work

The research on urban image in developed countries started earlier, and western scholars have carried out the exploration of urban image model from different perspectives in different periods. In the early days, the theoretical research on urban image carried out by scholars engaged in design practice was more prominent. The research on modern urban image has laid an important theoretical foundation for the development of modern urban image [4]. It can be analyzed that “architecture” should not only have the function of use but also emphasize the aesthetic significance and aesthetic value [5]. Literature [6] proposes the concept of “city image” and emphasizes that city image is obtained by perceiving the urban environment, which still belongs to the category of urban planning. It is emphasized that the city image needs not only to reflect the scientific and technological progress and the rationality of functional division but also to preserve the traditional historical context of the city. The new round of changes in the world city image is sweeping the world by western countries. Under the influence of this universal and standardized rational spirit, the traditional difference between cities has gradually become smaller. Each city is full of gray reinforced concrete forests. Bauhaus-style simple but impersonal buildings spread all over the world. There is no longer any difference between cities [7]. When a large number of city images have similar disadvantages, city designers and planners find that the personalization of city images can better enhance the image and spread the city image faster [8].

Literature [9] believes that many cities are in an important period of transition from the traditional urban model to the modern urban model. It is recommended to locate the overall style of the city and deduct the overall style to carry out urban construction. Literature [10] proposes a city visual recognition system. The following aspects should be considered in the construction of the project: comprehensive construction of urban information system, unified standardization of road signs, street signs, street lamps, garbage bins, unit signs, and the styles of stations in the city; creation of square culture; creation of hardware facilities for urban cultural landscapes; attention; unification of urban economic, social, cultural, and environmental benefits; establishment of influential large-scale cultural activities; change of mixed industrial and agricultural structures such as vegetable farms; creation of cultural groups with international influence [11]. Literature [12] studies the issue of urban image and urban cultural capital from the perspective of sociology, especially urban sociology, and in the sense of comprehensive disciplines recognizes the cultural symbols and symbolic meanings of urban image and proposes a transition from “running a city” to “marketing.” The operation of “city” and then “urban cultural capital” is the unification of social, cultural, and environmental benefits; the establishment of influential large-scale cultural activities; the transformation of mixed industrial and agricultural structures such as vegetable farms; and the creation of cultural groups with international influence. Literature [13] studies the issue of urban image and urban cultural capital from the perspective of sociology, especially urban sociology, and in the sense of comprehensive disciplines recognizes the cultural symbols and symbolic meaning of urban image and proposes a transition from “running a city” to “marketing.” The operation of “city” and then “urban cultural capital” is an innovation in the development of the core competitiveness of modern cities.

The city image design and its implementation are conducive to creating a city brand and increasing the city's comprehensive strength. In addition to promoting the construction of hardware facilities in the city, it also promotes the construction of software such as city culture, thus playing a positive role in the construction of socialist spiritual civilization, material civilization, and political civilization [14]. Urban image promotes the common development of urban culture and economy and promotes the comprehensive development of urban politics, culture, economy, and ideology [15]. The development model of urban construction will shift from purely economic growth and material production as the center to the balanced development mode of people-oriented and environmental sustainable development [16]. Carry out urban image design, combine the construction of urban spiritual civilization with the construction of urban image, make unified planning and implementation, and shape the image of urban characteristics [17]. In addition, urban image design can also improve the cultural, ideological, and moral level of residents, provide high-level, multiangle, and all-round education to urban residents, and promote the overall development of the city [18].

## 3. Nanchang VI Visual Image Recognition Model Based on Watson Perception Model

Nanchang VI visual image recognition model based on Watson perception model is constructed. Moreover, the model for measuring visual fidelity was proposed using ideas such as sensitivity and masking [19]. This perceptual model attempts to estimate the value of JND (just noticeable difference) between images. The main idea of this model is to evaluate the perceptibility of each coefficient obtained after an image is subjected to block DCT. Then, these evaluations are combined into a single parameter of perceptual distance *D*_wat_(*x*, *x*^*w*^), where *x* is the original image and *x*^*w*^ is some version of the image obtained after *x* is distorted.

Perceptual models can be based on many kinds of signal representations. The model adopts the block DCT transform; that is, the image is first divided into nonoverlapping 8 × 8 pixel blocks, and then the DCT transform is performed on each block, so that the image energy is concentrated on the low-frequency coefficients of each block. The Watson perceptual model is based on the block DCT transform and applies this model to JPEG compression. The perceptibility of the resulting quantization noise is assessed using the Watson model, making it possible to adapt the quantization step size to the characteristics of the image. However, the purpose of utilizing this model here is to evaluate and control the watermark embedding algorithm.

### 3.1. Sensitivity Characteristics

The sensitivity characteristic model defines a frequency sensitivity table **t**. Each entry *t*_*ij*_(0 ≤ *i*, *j* ≤ 7) in the table is approximately equal to the minimum value at which the corresponding DCT coefficient in the block cannot be resolved without masking noise (i.e., the corresponding change in the DCT coefficient produces exactly one unit of JND). Thus, a smaller value indicates that the human eye is more sensitive to this frequency. This sensitivity table is a parameter related to many parameters, including the resolution of the image and the distance of the observer to the image.

### 3.2. Luminance Masking Characteristics

Brightness adaptability means that if the average brightness of a 8 × 8 block of pixels is brighter, changing a DCT coefficient by a large amount goes unnoticed. For each patch, the model adjusts the sensitivity table *t* according to the magnitude of its DC component. The luminance masking threshold is

(1) $$\begin{array}{c} t_{ijk}^{L}=t_{ij}{\left(\frac{X_{00k}}{\bar{X}}\right)}^{a_{T}}, \end{array}$$

where *a*_*T*_ is a constant, and the recommended value is 0.649, *X*_00*k*_ represents the DC coefficient of the *k*-th pixel block of the original image, and $\bar{X}$ is the average value of all DC coefficients in the image. Additionally, $\bar{X}$ can be set to a constant that represents the desired image pixel value. Equation (1) shows that areas with higher brightness in the image can withstand larger changes without being noticed.

### 3.3. Contrast Masking Properties

The luminance contrast pair threshold *t*_*ijk*_^*L*^ is also affected by the contrast masking characteristics. Contrast masking properties (i.e., the energy of one frequency component makes changes in another frequency component less visible) result in a masking threshold matrix *s*_*ijk*_, which is defined as follows:

(2) $$\begin{array}{c} s_{ijk}=\max\left\{t_{ijk}^{L},{\left|X_{ijk}\right|}^{\beta_{ij}}•{\left(t_{ijk}^{L}\right)}^{1-\beta_{ij}}\right\}. \end{array}$$

Among them, *β*_*ij*_ is a constant between 0 and 1, and its value may be different for each frequency coefficient. For all *i* and *j*, *β*_*ij*_=0.7 is taken. The meaning of the final threshold value *s*_*ijk*_ is as follows. If the coefficient *X*_*ijk*_ in the block DCT changes by *s*_*ijk*_, a unit of JND will be generated. Usually, these thresholds are called Slacks.

### 3.4. General

To compare the original image **x** and the corresponding distorted image **x**^*w*^, the difference between the corresponding DCT coefficients is first calculated by *e*_*ijk*_=*X*_*ijk*_^*w*^ − *X*_*ijk*_. Then, the model scales these differences with the corresponding slack *s*_*ijk*_, so that the perceptual distance *d*_*ijk*_ of each item can be obtained:

(3) $$\begin{array}{c} d_{ijk}=\frac{e_{ijk}}{s_{ijk}}, \end{array}$$

where *d*_*ijk*_ represents the error of the *i*-th and *j*-th frequency components in the *k*-th block and the unit of this error is JND (its value represents a fraction or several times of the error of JND).

The individual errors calculated using (3) must be combined into a perceptual distance *D*_wat_(*x*, *x*^*w*^). Two forms of an integrated approach were employed. The first is to combine the errors of different pixel blocks, and the second is to combine the errors of different frequency components in the same pixel block. However, the exponents suggested for the *L*_*p*_-norm are the same for both errors. Therefore, the synthesis of these two forms can be combined into one equation as follows:

(4) $$\begin{array}{c} D_{\text{wat}}\left(x,x^{w}\right)={\left(\sum_{i,j,k}{\left|d_{ijk}\right|}^{p}\right)}^{1/p}. \end{array}$$

Among them, the value of *p* is 4.

Digital image scrambling is an image encryption technique. The scrambled image looks cluttered. It is difficult to restore the original image without knowing the type of scrambling transform used. At present, the scrambling techniques of digital images mainly include the following: Arnold transform, magic square, Hilbert curve, Conway game, Tangram algorithm, and IFS model.

Arnold transformation is a transformation prominent in Arnold's ergodic theory research, which is commonly known as cat face transformation. Its transformation formula is shown in formula (5).

We assume that there is a point (*x*, *y*) on the unit square, and the transformed point is (*x*′, *y*′).

(5) $$\begin{array}{c} \left[\begin{array}{c} x{}^{\prime }\\ y{}^{\prime } \end{array}\right]=\left[\begin{array}{cc} 1 & 1\\ 1 & 2 \end{array}\right]\left[\begin{array}{c} x\\ y \end{array}\right]\;\mathrm{mod}\;1. \end{array}$$

This transformation is a two-dimensional Arnold transformation. Applying the Arnold transform to a digital image can change the layout of image pixels by changing the pixel coordinates. If the digital image is regarded as a matrix, the transformed image will become messy. However, if you continue to use Arnold transformation, there will be an image that is the same as the original image; that is, Arnold transformation has periodicity.

The formula for Arnold scrambling for watermark images is shown as follows:

(6) $$\begin{array}{c} \left[\begin{array}{c} x{}^{\prime }\\ y{}^{\prime } \end{array}\right]=\left[\begin{array}{cc} 1 & 1\\ 1 & 2 \end{array}\right]\left[\begin{array}{c} x\\ y \end{array}\right]\;\mathrm{mod}\;N. \end{array}$$

Among them, (*x*, *y*) is the coordinate point on the watermark image, (*x*′, *y*′) corresponds to the coordinate point of the scrambled image, and N is the pixel height or width of the watermark image.

Figure 1 shows the original image (a) and the image after 15 Arnold scrambling transformations (b).

The adaptive selection process of the embedded region is as follows. Firstly, the video image is divided into nonoverlapping blocks, each block is DCT transformed in turn to obtain the DCT coefficient matrix *X* of each block, and the DCT coefficients are arranged in the order of “zigzag.” Then, it is divided into brightness blocks according to the value of the DC coefficient, and then the details of the image are classified according to the energy of the DCT AC coefficient.

Here, the energy of the DCT AC coefficient is denoted by *E*_*AC*_; that is,

(7) $$\begin{array}{c} E_{AC}=\mathrm{lg}\left(\sum_{k=1}^{N}X_{k}^{2}\right). \end{array}$$

The logarithmic operation in formula (7) is to narrow the range of values and maintain monotonicity. For each DCT coefficient block, if its energy *E*_*AC*_ is less than a given threshold, the corresponding image block is a low-detail area; otherwise, it is a high-detail area.

The proposed watermark embedding algorithm embeds the watermark information into the DCT low-frequency coefficients of the luminance block in the I-frame. The main reasons are as follows:

1. The low-frequency coefficients concentrate most of the energy of the signal and belong to the important components in the signal. However, embedding the watermark into these coefficients is robust enough, and combined with the human visual system model, appropriate modification of the low-frequency coefficients can achieve a balance between imperceptibility and robustness.
2. Generally, the low-frequency coefficient has a larger value, and the impact on the image quality after embedding the watermark information is small, which is beneficial to ensure invisibility.
3. Embedding the watermark information into the high-frequency coefficients can well ensure the invisibility of the watermark. However, at the same time, signal processing methods such as lossy compression, filtering, and adding noise are also easy to remove the watermark, and the robustness is poor.

The watermark embedding algorithm is as follows:

Step 1: The algorithm generates a watermark signal. The algorithm uses the Arnold image scrambling technology to scramble the watermarked image to generate the watermark signal W.
Step 2: The algorithm performs MPEG-4 encoding on the original video and performs 16 × 16 macroblock division on the I-frame.
Step 3: The algorithm performs 8 × 8 block division on the macroblock and performs DCT transformation and quantization on the four 8 × 8 luminance blocks in the macroblock.
Step 4: The algorithm determines the high-detail and high-brightness watermark information embedding areas. The algorithm calculates the energy *E*_*AC*_ of the 8 × 8 luminance block according to equation (7). For each block of DCT coefficients, if *E*_*AC*_ is less than a predetermined interval value *T*_*D*_, the corresponding block is divided into low-detail regions; otherwise, the corresponding block is divided into high-detail regions. Similarly, compare the DC component of the DCT coefficient block with the given threshold *T*_*M*_*T*_*M*_; if the value is greater than that, it is a high-brightness area; otherwise, it is a low-brightness area. The selection of TD and TM should fully consider the two factors of video quality and robustness.
Step 5: The algorithm obtains the polarity *P*_*i*_ of the 8 × 8 luminance DCT block according to the formula (8) for the block that needs to be embedded with the watermark.
  (8) $$\begin{array}{c} P_{i}=\left\{\begin{array}{cc} 1, & \left|X_{i}\right|>\left|s\cdot X_{0}\right|,\\ 0, & \text{other,} \end{array}\right. \end{array}$$
where *s* is a constant, which represents the scaling factor of the DC coefficient. *X*_*i*_ represents several continuous low-frequency AC coefficients of the 8 × 8DCT block, *X*_0_ represents the DC coefficient, and their values are shown in the following equation:
  (9) $$\begin{array}{c} \left\{\begin{array}{c} X_{i}=X_{i}•Q_{i},\\ X_{0}=X_{0}•Q_{0}, \end{array}\right. \end{array}$$
where *Q*_*i*_ represents the quantization coefficient in the MPEG-4 quantization matrix.
Step 6: The algorithm calculates the slack *S*_*i*_ of the coefficients that need to be modified in the current block according to equations (1) and (2).
Step 7: The algorithm embeds watermark information according to the following formula:
  (10) $$\begin{array}{c} X_{i}^{w}=\left\{\begin{array}{cc} X_{i}+S_{i}, & P_{i}\neq w_{i}Ç\text{Ò }w_{i}=1,\\ X_{i}-S_{i}, & P_{i}\neq w_{i}Ç\text{Ò }w_{i}=0,\\ X_{,i} & P_{i}=w_{i}, \end{array}\right. \end{array}$$

where *X*_*i*_^*w*^ and *X*_*i*_ are the DCT coefficients before and after embedding the watermark, respectively, *S*_*i*_ is the slack degree corresponding to the modified coefficients, and they satisfy the following relationship:

(11) $$\begin{array}{c} \left|X_{i}+S_{i}\right|-\left|s•X_{0}\right|\geq \varepsilon ,\\ \left|s•X_{0}\right|-\left|X_{0}-S_{i}\right|\geq \varepsilon , \end{array}$$

where *ε* is a suitable positive number to ensure the robustness to MPEG compression. In order to ensure the video image quality, *S*_*i*_ should be properly adjusted to make it the same number as *X*_*i*_.

The watermark extraction algorithm is relatively simple, and it does not need to utilize the original image.

**Step 1 .**

The algorithm decodes the I-frame to obtain the 16 × 16 macroblock and 8 × 8 luminance block information.

**Step 2 .**

The algorithm calculates the energy of the 8 × 8 luminance block according to the formula (7) and determines the high luminance and high-detail area according to the DC component, which is the image block with a watermark information.

**Step 3 .**

The algorithm uses equation (12) to get the watermark bit.

(12) $$\begin{array}{c} w_{i}=\left\{\begin{array}{cc} 1, & \left|X_{i}\right|>\left|s•X_{0}\right|,\\ 0, & \left|X_{i}\right|\leq \left|s•X_{0}\right|. \end{array}\right. \end{array}$$

**Step 4 .**

The algorithm repeats the above steps until all the watermark information is extracted.

The programming environment of this experiment is Visual *C*++ 2008, and the Xvid MPEG-4 codec model is used. Due to the particularity of the Arnold transform, the watermark image adopts a binary image with equal length and width of 32 × 32. The test video uses the standard video sequence: bus_cif.yuv, foreman_cif.yuv, coastguard_cif.yuv. The parameters of the three videos are shown in Table 1.

#### 3.4.1. Imperceptibility Analysis

The objective evaluation of image quality refers to the use of one or some quantitative parameters and indicators to describe the image quality. It has important value in image compression, image watermarking, and other applications, and it is an important indicator to measure the performance of different algorithms. The most common image evaluation criteria are peak signal-to-noise ratio (PSNR) and mean square error (MSE). In this paper, the imperceptibility is objectively judged by calculating the peak signal-to-noise ratio (PSNR). The calculation formula of PSNR is shown in formula (14):

(13) $$\begin{array}{c} \text{PSNR}=10\;\log_{10}\left(\frac{255^{2}}{MSE}\right). \end{array}$$

Among them, MSE is the mean square error, and its calculation formula is shown in the following formula:

(14) $$\begin{array}{c} \text{MSE}=\frac{1}{MN}\sum_{x=1}^{M}\sum_{y=1}^{N}{\left[f{}^{\prime }\left(x,y\right)-f\left(x,y\right)\right]}^{2}. \end{array}$$

Among them, *f*(*x*, *y*) is the original video data, and *f*′(*x*, *y*) is the processed video data. *M* and N are the width and height of the encoded video, respectively.

Under normal circumstances, it is generally believed that the PSNR of 30 db is difficult for the human eye to distinguish the difference between the two images before and after processing, and the larger the PSNR value, the better the imperceptibility of the video.

Figure 2 is the original video image without the watermark embedded, and Figure 3 is the corresponding video image with the watermark embedded. From the subjective visual observation, there is almost no difference.

Table 2 shows the peak signal-to-noise ratio (PSNR) of some I-frame images in each video sequence after encoding, that is, after embedding the watermark.

It can be seen from the experimental results that the algorithm in this paper is satisfactory in the experimental effect of imperceptibility.

#### 3.4.2. Robustness Analysis

For each observer, the fidelity of the extracted digital watermark depends on their subjective views. This is related to many factors of the observer, such as experience and sensitivity to images. Therefore, subjective observation is arbitrary. Therefore, we need to objectively measure the similarity between the extracted watermark and the original watermark by quantitative analysis.

In this paper, the normalized correlation coefficient (NC) is used to objectively judge the similarity between the extracted watermark and the original watermark. The calculation formula of the normalized correlation coefficient of the watermark is shown as follows:

(15) $$\begin{array}{c} NC=\frac{\sum \sum w\left(m,n\right)w{}^{\prime }\left(m,n\right)}{\sqrt{\sum \sum w^{2}\left(m,n\right)}\sqrt{\sum \sum w^{\prime 2}\left(m,n\right)}}. \end{array}$$

Table 3 shows that the robustness of the watermarking algorithm in this paper is objectively evaluated by calculating the normalized correlation coefficient of the watermarked image.

From the data in Table 3, it can be known that the algorithm in this paper has strong robustness to MPEG-4 encoding and frame deletion attacks, and it can basically completely extract the watermark information. For the attack of randomly deleting video frames, the algorithm in this paper only embeds the watermark information in the I-frame. However, the I-frame is often used as the starting frame of a scene, and the P and B frames are both predicted from the I-frame during video decoding. Therefore, the I-frame is not allowed to be deleted from the video stream, so the algorithm in this paper has strong robustness to frame deletion attacks. It can also be seen from the table that the algorithm in this paper has poor robustness to lossy compression and needs further improvement.

Embedding the watermark information in the low-frequency coefficients in DCT can not only ensure the robustness of the watermark but also meet the imperceptibility. In this section, by choosing the second scheme, the watermark is embedded in the encoding process, and the watermark is extracted in the decoding process. The specific process is shown in Figure 4.

The principle of watermark embedding is shown in Figure 5.

The embedding process is:

Step 1: The algorithm inputs the watermark information and generates a key according to the watermark content.
Step 2: The algorithm reads the original video sequence, divides it into 16 × 16 nonoverlapping macroblocks, performs DCT transformation on the divided data, and quantizes it in an intraframe manner.
Step 3: The algorithm performs AC/DC prediction on the quantized macroblock, further compresses it, and then restores the corresponding coefficients according to the different prediction modes.
Step 4: The algorithm selects four 8 × 8 luminance blocks of each macroblock in the video I-frame and extracts three regions *S*_1_, *S*_2_, *S*_3_ from the medium- and low-frequency coefficients of each luminance block, as shown in Figure 6.
  (a) The algorithm calculates the energies *E*_1_, *E*_2_, *E*_3_ of the three selected regions in Figure 7, respectively, according to the following formula:
    (16) $$\begin{array}{c} E_{k}=\sum_{i,j\in S_{k}}\left|X_{ij}\right|\;k=1,2,3. \end{array}$$
  (b) The algorithm sorts the energies of the three regions to get *E*_high_, *E*_mid_, *E*_low_.
  (c) The algorithm calculates the energy average *E*_avg_ and the energy range *E*_range_ of the three regions according to (17) and (18), respectively.
    (17) $$\begin{array}{c} E_{\text{avg}}=\frac{1}{3}\left(E_{\text{high}}+E_{\text{mid}}+E_{\text{low}}\right), \end{array}$$
    (18) $$\begin{array}{c} E_{\text{range}}=E_{\text{high}}-E_{\text{low}}. \end{array}$$
  (d) The algorithm uses (19) to change *E*_mid_ into *E*_mid_′.
    (19) $$\begin{array}{c} E_{\text{mid}}^{\prime }=E_{\text{avg}}+\alpha E_{\text{range}}*{\left(-1\right)}^{w_{i}}, \end{array}$$
  where *α* is the parameter that controls the perturbation amplitude, *w*_*i*_ represents the watermark bit, and *w*_*i*_ ∈ {0,1}.
  (e) The algorithm calculates the average modification magnitude according to the following equation:
    (20) $$\begin{array}{c} T=\frac{E_{\text{mid}}^{\prime }-E_{\text{mid}}}{3}. \end{array}$$
  (f) The algorithm modifies the DCT coefficients in the *S*_mid_ region according to the following rules. Among them, *X*_*ij*_ is the DCT coefficient before modification, *X*_*ij*_^*w*^ is the modified DCT coefficient, and *i*, *j* ∈ *S*_mid_.
  (1) If *w*_*i*_=0 and *E*_mid_ ≥ *E*_mid_′ or *W*_*i*_=1 and *E*_mid_ < *E*_mid_′, the DCT coefficient remains unchanged; that is,
    (21) $$\begin{array}{c} X_{ij}^{w}=X_{ij}. \end{array}$$
  (2) If *w*_*i*_=0, *E*_mid_ < *E*_mid_′, and *X*_*ij*_ ≥ 0 are established, the following formula is established:
    (22) $$\begin{array}{c} X_{ij}^{w}=X_{ij}+T. \end{array}$$
  (3) If *w*_*i*_=0, *E*_mid_ < *E*_mid_′, and *X*_*ij*_ < 0 are established, the following formula is established:
    (23) $$\begin{array}{c} X_{ij}^{w}=X_{ij}-T. \end{array}$$
  (4) If *w*_*i*_=1, *E*_mid_ ≥ *E*_mid_′, and *X*_*ij*_ ≥ 0 are established, the following formula is established:
    (24) $$\begin{array}{c} X_{ij}^{w}=X_{ij}-T. \end{array}$$
  If the above formula makes *X*_*ij*_^*w*^*∗X*_*ij*_ < 0, then *X*_*ij*_^*w*^=0.
  (5) If *w*_*i*_=1, *E*_mid_ ≥ *E*_mid_′, and *X*_*ij*_ < 0 are established, the following formula is established:
    (25) $$\begin{array}{c} X_{ij}^{w}=X_{ij}+T. \end{array}$$
  If the above formula makes *X*_*ij*_^*w*^*∗X*_*ij*_ < 0, then *X*_*ij*_^*w*^=0.
Step 5: The algorithm loops through the above operations for all macroblocks until all watermark information is embedded.

Watermark extraction is the inverse process of embedding. The algorithm in this section directly uses the MPEG-4 video containing watermark information for partial decoding to obtain the quantized video data and extracts the watermark information from it. Its process is shown in Figure 7.

Step 1: The algorithm performs VLD decoding on the MPEG-4 video and obtains the DCT coefficients after I-frame quantization.
Step 2: The algorithm selects the three regions shown in Figure 7 and calculates the energy balance value EB according to the following formula:
  (26) $$\begin{array}{c} EB=EH-EL\\ =2\alpha *{\left(-1\right)}^{w_{j}+1}*\left(E_{\text{high}}-E_{\text{low}}\right). \end{array}$$
In the formula, there are
  (27) $$\begin{array}{c} EH=E_{\text{high}}-E_{\text{mid}},\\ EL=E_{\text{mid}}-E_{\text{low}}. \end{array}$$
If *EB* ≥ 0, then *w*_*i*_=1; otherwise, *w*_*i*_=0.
Step 3: The algorithm uses the key to extract all the watermark information and uses the majority principle to compress the extracted watermark sequence to obtain the original watermark sequence.
Step 4: The algorithm restores the watermark information content.

Taking the waterfall video sequence as an example for analysis, Table 4 gives the peak signal-to-noise ratio (PSNR) of some I-frame images in each video sequence after encoding, that is, after embedding the watermark.

Since the PSNR value is above 30 dB, it is difficult for the human eye to distinguish the difference between the two images before and after processing. It can be seen from the experimental results that the algorithm in this paper is satisfactory in the experimental effect of imperceptibility.

## 4. Conclusion

The establishment of the visual recognition system is the most intuitive and accurate form of visual communication, and it becomes a bridge and link to enhance the city's image, spread the city's culture, and build attractiveness to the public. The influence of people's ideas, emotions, and consciousness in the spiritual and cultural field determines the establishment of the visual recognition system to enhance the core competitiveness of the overall city image with its unique and attractive form of expression. At present, China's urban image construction currently has problems such as lack of integrity, standardization, stability, and identification. The establishment of the city image visual identification system is based on the corporate image identification system (CIS) and extended. This paper combines the Watson visual perception model to implement the Nanchang VI visual image recognition design and improve the communication effect of the urban VI visual image. Finally, this paper verified the reliability of the method in this paper through the study of multiple sets of data.

## Figures and Tables

**Figure 1:** Comparison of Arnold images before and after scrambling: (a) original image and (b) scrambling the transformed image.

**Figure 2:** Original video image.

**Figure 3:** The video image after embedding the watermark.

**Figure 4:** Watermark embedding and extraction process.

**Figure 5:** Schematic diagram of watermark embedding.

**Figure 6:** Three selection areas for an 8 × 8 block.

**Figure 7:** Schematic diagram of watermark extraction.

**Table 1:** Experimental video parameters.

Video sequence	Bus	Foreman	Coastguard
Video length	150 frames	300 frames	300 frames
Frame size	352 × 288	352 × 288	352 × 288

**Table 2:** Peak signal-to-noise ratio of I-frame image after embedding watermark.

PSNR video sequence	1st I-frame (dB)	2nd I-frame (dB)	3rd I-frame (dB)	4th I-frame (dB)
Bus	39.5011	40.3697	39.1072	39.5415
Foreman	40.2687	37.4912	39.895	39.2688
Coastguard	39.2284	39.1072	39.5011	38.5012

**Table 3:** Robustness analysis of watermarking algorithm.

Video sequence attack type	Foreman	Bus	Coastguard
MPEG-4 encoding	1.00000	0.999698	1.00000
Lossy compression	0.553278	0.607212	0.692759
Median filtering	0.787396	0.755581	0.797496
Noise	0.763459	0.762449	0.835169
Frame delete	1.00000	1.00000	1.00000

**Table 4:** Peak signal-to-noise ratio (dB) of I-frame image after embedding watermark.

Video sequence frame number	Waterfall	Foreman	Coastguard
Frame 1	39.693	39.8344	38.9052
Frame 26	39.0567	41.3393	35.6126
Frame 51	39.0567	39.5819	34.3905
Frame 76	39.0365	39.8647	33.5017
Frame 101	39.0668	37.9356	33.4815
Frame 126	38.986	41.5312	33.6229
Frame 151	38.9759	38.178	35.8954
Frame 176	38.9456	38.6325	34.6632
Frame 201	38.9355	38.1376	35.8752
Frame 226	37.9053	39.3395	35.8752

## Data Availability

The labeled dataset used to support the findings of this study is available from the corresponding author upon request.
